The article "Effects of Different Surgical Procedures on the Therapeutic Effects, Prognosis, and Major Complications of Acetabular Fractures in the Elderly of China: A Systematic Review and Meta-Analysis" was published in 2022. Journal: Comput Math Methods Med.

# Effects of Different Surgical Procedures on the Therapeutic Effects, Prognosis, and Major Complications of Acetabular Fractures in the Elderly of China: A Systematic Review and Meta-Analysis

**DOI:** 10.1155/2022/9249920

**Published:** 2022-08-18

**Authors:** Lei Wen, Kun Liu, Ge Chen, Jianhua Ji, Changshun Chen, Zhong Chen

**Affiliations:** ^1^Department of Orthopaedic and Trauma Surgery, Affiliated Hospital of Yunnan University, Kunming, Yunnan Province 650000, China; ^2^Department of Anesthesiology, The First Affiliated Hospital of Kunming Medical University, Kunming City, Yunnan Province 650000, China

## Abstract

**Objective:**

Different surgical approaches were systematically evaluated to provide an evidence-based medical rationale for the application and promotion of acetabular fractures in the elderly of China.

**Methods:**

Randomized controlled trials (RCT) of different surgical methods in the treatment of elderly acetabular fractures were searched in the PubMed, EMBASE, ScienceDirect, Cochrane Library, China Knowledge Network Database (CNKI), China VIP Database, Wanfang Database, and China Biomedical Literature Database (CBM). The search time threshold was set from the time the database was created to the current time. Investigators obtained data independently, and the bias risk of each included writing was reviewed using the Cochrane Manual 5.1.0 criterion. The meta data was analyzed using RevMan 5.4 statistical package.

**Results:**

6 RCT articles were included in the end. A total of 445 samples were analyzed by meta. All the six RCT literatures included in this meta-analysis reported the baseline status of patients, only 3 RCT mentioned “random assignment” without any explanation, and the rest did not mention “random” information. The five studies included all gave detailed intervention measures. The number and reasons of blind method and lost follow-up or withdrawal were not described in detail in 6 RCT articles. Through the meta-analysis excellent and good rate between the experimental group and the control group through 6 RCT studies, the heterogeneity test results were chi^2^ = 6.11, df = 4, P = 0.19 > 0.05, and I^2^ = 35%, without obvious heterogeneity at *Z* = 2.68 and *P* = 0.007. These results suggested that the total hip arthroplasty application has the same excellent rate as other surgical treatment methods, indicating that total hip arthroplasty has a significant effect on the treatment of elderly acetabular fractures. Through the meta-analysis hip-joint function score, the heterogeneity test results were chi^2^ = 56.16, df = 4, *P* < 0.00001, and *I*^2^ = 93%, with obvious heterogeneity. The great difference was discovered in hip function score between total hip arthroplasty and other surgical methods, showing that total hip arthroplasty can greatly improve hip-joint function. Then, the incidence of hip complications between the experimental cases and the control cases was calculated by meta. The heterogeneity test results were chi^2^ = 3.17, df = 4, *P* = 0.53 > 0.05, and *I*^2^ = 0%, without remarkable heterogeneity at *Z* = 3.05 and *P* = 0.002. This demonstrated that a significant difference was observed in the complication incidence, indicating that total hip arthroplasty displayed a lower incidence of hip-joint functional complications.

The article "Effects of Different Surgical Procedures on the Therapeutic Effects, Prognosis, and Major Complications of Acetabular Fractures in the Elderly of China: A Systematic Review and Meta-Analysis" was published in 2022. Journal: Comput Math Methods Med.

**Conclusion:**

Total hip arthroplasty has a good prognosis and a low complication rate in the treatment of acetabular fractures in the elderly. However, more studies and longer follow-ups are needed to further validate the findings of this study.

## 1. Introduction

An acetabular fracture is a break in the socket portion of the “ball-and-socket” hip joint. In the past, acetabular fractures were treated conservatively. Conservative treatment involves prolonged bed rest and many complications (e.g., early joint degeneration or avascular necrosis of the femoral head). It often fails to restore the matching relationship between the femoral head and the acetabulum and therefore has a very poor outcome. With the continuous improvement of diagnosis and treatment technology and the emergence of new internal fixation equipment, open reduction and internal fixation have become the gold standard for the treatment of displaced acetabular fractures [1]. As there are many factors that affect the effect of treatment, even if treated by experienced specialists, there may still be some postoperative complications, affecting the long-term effect. The common complications affecting joint function after acetabular fracture are traumatic arthritis, osteonecrosis of the femoral head, heterotopic ossification, nerve injury, and so on.

Traumatic arthritis is the most common complication after operation of medullary acetabular fracture with an incidence of 12%-57% [2], which occurs in all types of acetabular fractures. Poor reduction is the main factor leading to traumatic arthritis [3]. When traumatic arthritis progresses with severe pain and dysfunction, surgical treatment is often needed. The popular surgical approaches are hip arthroplasty and hip replacement, which are often not accepted by patients because of the problems of hip fixation after hip fusion [4]. Total hip arthroplasty (THA) is an ideal method for the treatment of acetabular fractures, but whether fresh acetabular fractures need one-stage total hip replacement is still controversial [5, 6]. Its indications should be strictly grasped. Petohazi et al. used one-stage total hip arthroplasty to treat acetabular posterior column fractures with femoral head and neck fractures with satisfactory results [7–9]. At present, there are few articles on meta-analysis of acetabular fractures in the elderly with different surgical methods. In view of the small number of patients included in the individual articles and their age, the meta-analysis is again carried out in this paper, taking into account the high-quality relevant literature published in recent years, both nationally and internationally. In this paper, meta-analysis was used to compare the treatment effects, prognosis, and main complications of different surgical methods in the treatment of acetabular fractures in the elderly, in order to provide options for clinicians to choose a more optimized and more suitable treatment plan for patients.

The article "Effects of Different Surgical Procedures on the Therapeutic Effects, Prognosis, and Major Complications of Acetabular Fractures in the Elderly of China: A Systematic Review and Meta-Analysis" was published in 2022. Journal: Comput Math Methods Med.

## 2. Research Content and Methods

### 2.1. The Sources and Retrieval Methods of Documents

Randomized controlled trials (RCT) of different surgical methods in the treatment of elderly acetabular fractures were searched in the Cochrane Library, PubMed, Embase, OVID, China Knowledge Network Database (CNKI), Wanfang Database, China Biomedical Literature Database (CBM), and VIP Central Database (VIP). Chinese search words were “total hip arthroplasty, traditional surgery, pelvic fracture, acetabular fracture, randomized controlled trial,” etc.; manual search was conducted of references and grey literature included in the literature in order to find potential studies that meet the inclusion criteria of this system evaluation. The search time threshold was set from the time the database was created to the current time and the language is limited to Chinese.

### 2.2. Literature Inclusion Criteria and Exclusion Criteria

#### 2.2.1. Literature Inclusion Criteria

The literature inclusion criteria are as follows: (1) the type of research was a randomized controlled trial (RCT) and the language is Chinese only; (2) the intervention subjects were patients with pelvic and acetabular fractures diagnosed clearly, regardless of age, sex, race, or region; (3) the intervention measures were total hip arthroplasty and other operations; (4) the observation indexes included operation time, intraoperative blood loss, postoperative complications, hospital stay, clinical effect, incision length, drainage volume, extubation time, blood transfusion volume, Matta score, Harris score, imaging results, Merled score, and so on.

#### 2.2.2. Literature Exclusion Standard

The literature exclusion criteria are as follows: (1) retrospective studies, cohort studies, case reports, etc.; (2) the studies with incomplete results; (3) the research with a too small sample size (less than 20 cases); (4) repeated studies: repeated reports from the same team.

The article "Effects of Different Surgical Procedures on the Therapeutic Effects, Prognosis, and Major Complications of Acetabular Fractures in the Elderly of China: A Systematic Review and Meta-Analysis" was published in 2022. Journal: Comput Math Methods Med.

### 2.3. Quality Evaluation and Data Extraction

The quality was evaluated by two scholars with reference to the bias risk assessment criteria of the Cochrane Collaboration Network, including the following aspects: the generation of random methods, the concealment of allocation schemes, whether participants are blind, data integrity of results, selective reporting, and other sources of bias [10]. The documents were independently extracted and cross-checked by two evaluators. When there were differences between the two, an agreement was reached through consultation. It included the author(s), published time, sample size, treatment method, curative effect evaluation method, and so on.

### 2.4. Statistical Processing

The standardized mean difference (SMD) with Hedges' *g* was chosen as the measure of the effect. The effect size was calculated using a random-effect model with a restricted maximum-likelihood (REML) and considered a large, moderate, and small effect with respect to the SMD values of 0.8, 0.5, and 0.2, respectively. The heterogeneity among the studies included in a meta-analysis was assessed using Cochrane's *Q*, tau-squared, and *I*-squared (*I*^2^). Cochrane's *Q* test quantifies total variance and generates a *P* value that determines that heterogeneity is present. Tau-squared indicates the true variance that is the between-study variance, while *I*^2^ represents the percentage of the total variance that is due to the true variance. The degree of heterogeneity is said to be low, moderate, and high, with *I*^2^ values of 25%, 50%, and 75%. RevMan 5.4 software was adopted for meta-analysis. HR and its 95% CI were employed as effect analysis statistics for OS and PFS, and risk ratio and 95% CI were employed as effect analysis statistics for binary variables. *P* and *I*^2^ values in heterogeneity test results were adopted to determine whether there was statistical heterogeneity among the results. *P* > 0.10 and *I*^2^ < 50% indicated that there was no statistical heterogeneity among the research results, and a fixed-effect model was used for combined analysis. *P* ≤ 0.10 and *I*^2^ ≥ 50% indicated statistical heterogeneity among the research results, and a random-effect model was adopted for combined analysis. The test level of meta-analysis was set as *α* = 0.05. Eggers' test was used to examine the funnel plot asymmetry. Whenever this test was significant with a *P* value of less than 0.1, we used the trim and fill method to correct the funnel plot and adjust the effect size for potential publication bias.

The article "Effects of Different Surgical Procedures on the Therapeutic Effects, Prognosis, and Major Complications of Acetabular Fractures in the Elderly of China: A Systematic Review and Meta-Analysis" was published in 2022. Journal: Comput Math Methods Med.

## 3. Results and Analysis

### 3.1. The Results of Literature Retrieval and the Basic Situation of Literature Inclusion

2431 papers were retrieved through computer database retrieval; 242 papers were obtained after excluding duplicate studies; 105 papers were obtained by preliminary reading of the titles and abstracts of the papers, excluding unrelated studies, reviews, case reports, and noncontrol literatures; 21 articles were initially included; and then, 15 articles with incomplete data and no main outcome indicators were read carefully. In the end, 6 RCT [11–16] were included in the current analysis (Table 1).

### 3.2. Evaluation of the Methodology Quality Included in the Literature

All the six RCT literatures included in this meta-analysis reported the baseline status of patients, only 3 RCT mentioned “random assignment” without any explanation, and the rest did not mention “random” information. The five studies included all gave detailed intervention measures. The number and reasons of blind method and lost follow-up or withdrawal were not described in detail in 6 RCT articles. The proportion of various biases included in the study is shown in Figure 1, and the study quality evaluation and risk assessment are included in Figure 2.

### 3.3. Meta-Analysis Result

#### 3.3.1. Excellent and Good Rate

Through the meta-analysis excellent and good rate among 6 RCT studies, heterogeneity tests were chi^2^ = 6.11, df = 4, *P* = 0.19 > 0.05, and *I*^2^ = 35%, without no obvious heterogeneity at *Z* = 2.68 and *P* = 0.007. The results were considered that the total hip arthroplasty has the same excellent rate as other surgical treatment methods. Significant difference was found, indicating that total hip arthroplasty in the treatment of elderly acetabular fractures was effective (Figure 3).

#### 3.3.2. Hip-Joint Function Score

Through the meta-analysis hip-joint function score between the experimental group and the control group of 6 RCT studies, the heterogeneity test suggested chi^2^ = 56.16, df = 4, *P* < 0.00001, and *I*^2^ = 93%, with obvious heterogeneity. The results implied there was obvious differences in the hip-joint function score, meaning that total hip arthroplasty was able to greatly enhance the hip-joint function (Figure 4).

#### 3.3.3. Complication Incidence

Overall, 445 samples from 6 RCT studies were included. The incidence of hip complications between the experimental group and the control group was analyzed by meta-analysis. The heterogeneity test results were chi^2^ = 3.17, df = 4, *P* = 0.53 > 0.05, and *I*^2^ = 0 without obvious heterogeneity at *Z* = 3.05 and *P* = 0.002. This meant there were markable differences in the complication incidence, indicating that total hip arthroplasty has less incidence of hip-joint functional complications. Due to the small number of literatures included in the analysis, it was not suitable to make a funnel chart, but the analysis may have a certain degree of publication bias (Figure 5).

The article "Effects of Different Surgical Procedures on the Therapeutic Effects, Prognosis, and Major Complications of Acetabular Fractures in the Elderly of China: A Systematic Review and Meta-Analysis" was published in 2022. Journal: Comput Math Methods Med.

## 4. Discussion

The hip joint is the largest and most important weight-bearing joint in the human body. The treatment of acetabular fractures is a great challenge for orthopedic surgeons due to the special anatomical position of the acetabulum, its irregular anatomical form, and changing fracture types [17, 18]. With the average life expectancy of human beings having increased significantly, the proportion of the elderly population has greatly increased [19]. A few studies have shown that the proportion of elderly people over 60 years old in patients with acetabular fractures increased by 1.4 times from 1980 to 2007 [20]. In elderly patients with acetabular fractures, the difficulty of treatment is magnified by the complex fracture pattern, the poor biomechanical properties of the bone, and the number of underlying diseases [21, 22]. In the past, due to the limitations of the development of medical technology, many elderly patients with acetabular fractures had to undergo conservative treatment, which often required long-term brake or bed rest, which would lead to the decline of the function of the bone and muscle system [23].

In the 1860s, Yu et al. [24] took the lead in proposing surgical treatment of acetabular fractures in the elderly, which was supported and imitated by many scholars, and achieved good results. The scholars performed statistical classification on 120 elderly patients with acetabular fractures [25]. As the patients' age increased, their prognosis became worse and worse, but they still had a high excellent and good rate. Ali et al. reported 21 cases of elderly acetabular fractures involving the tetragonal area [26]. Although the anatomic reduction rate was only 52.4%, the SF-12PCS and Harris scores were satisfactory after an average follow-up of 4.2 years. ElSherif and Abonnour reported that 18 elderly patients with acetabular fractures were treated with open reduction and internal fixation [27]. The average follow-up was 31 months. The results showed that the Harris score was 90. Only one patient needed two-stage total hip arthroplasty because of aseptic necrosis of the femoral head. Many studies have demonstrated that although the rate of anatomical repositioning in elderly patients with acetabular fractures is lower than that in younger patients, long-term functional outcomes remain satisfactory and only a minority of patients require a repeat total hip replacement. Therefore, for elderly patients with acetabular fractures with obvious displacement, except for some special types of fractures that need one-stage total hip arthroplasty, open reduction and internal fixation should be the first choice [28]. In order to reduce the incidence of postoperative hip pain, traumatic osteoarthritis, and failure of internal fixation, acetabular fracture surgery should achieve hip white anatomical reconstruction and maintain concentric reduction of the hip joint [29].

The article "Effects of Different Surgical Procedures on the Therapeutic Effects, Prognosis, and Major Complications of Acetabular Fractures in the Elderly of China: A Systematic Review and Meta-Analysis" was published in 2022. Journal: Comput Math Methods Med.

Acetabular fractures are generally poor, and the emergency surgery is not recommended [30]. The delayed operation easily forms heterotopic ossification and fixation deformity, and fixation is difficult. Therefore, when the vital signs permit, the fracture should be treated as soon as possible, in which the best time is 3-7 days [31]. For old acetabular fractures that have been more than 3-4 months, the opportunity for surgical reduction is basically lost and total hip arthroplasty may be more effective [32, 33]. Acetabular fractures are intra-articular fractures, which should follow the principles of anatomical reduction, effective internal fixation, and early functional exercise. For acetabular fracture with posterior dislocation of the hip joint, closed reduction of the hip joint should be performed first, followed by acetabular reduction. The acetabulum is a complex geometry with various curves and radians. In order to achieve strong internal fixation, there are different internal fixation methods and internal fixation devices for different types of fractures [34, 35]. The main results are as follows: (1) Steel wire internal fixation is suitable for fractures in which the fracture line extends to the large notch of the ischium, including partial posterior column, horizontal, and double column fractures, especially for elderly patients with osteoporosis; the operation is relatively simple, but the strength is poor; it is often used in combination with other internal fixation methods. (2) Reconstruction plate internal fixation: the reconstruction plate can be well molded according to the anatomical morphology of the acetabulum, and the biomechanics is stable, but accurate prebending is needed. There is a possibility of postoperative traumatic arthritis caused by screw penetration into the joint cavity and fracture displacement during screw compression. (3) Locking compression plate internal fixation system: the overall stability between the plates and nails of the locking compression plate internal fixation system is equivalent to the internal fixation bracket, with high fixation strength, low shaping requirements, and simple fixation of the posterior wall, and it allows the steel plate to leave the bone surface for fixation. There is no need to peel off the periosteum or expose more soft tissue during the operation, which can effectively protect the blood flow of the fracture end and reduce the occurrence of heterotopic ossification after operation. (4) Memory alloy three-dimensional internal fixation system for acetabular fractures. (5) Percutaneous screw fixation: percutaneous screw fixation is often combined with fluoroscopic navigation. This new method combines computer image processing and visualization technology with clinical surgery in the form of interactive image navigation. Using infrared devices on the patient and surgical instruments, the position of the patient's bones and the position of the surgical instruments can be determined, providing real-time spatial position and movement of the surgical instruments and visualising this information to the operator to complete the operation accurately. At present, there are two-dimensional perspective navigation and three-dimensional perspective navigation. Percutaneous screw fixation under the guidance of two-dimensional perspective navigation for the treatment of acetabular fractures has been accepted by more and more orthopedic surgeons and has been popularized in a certain range. The more visual and intuitive three-dimensional perspective navigation is a new technology, which can display images of the hip joint on the sagittal, coronal, and cross-sections at the same time on the display. Although it is still in the exploratory stage, it has broad application prospects [36].

The article "Effects of Different Surgical Procedures on the Therapeutic Effects, Prognosis, and Major Complications of Acetabular Fractures in the Elderly of China: A Systematic Review and Meta-Analysis" was published in 2022. Journal: Comput Math Methods Med.

Artificial hip replacement began in the 1940s [37]. According to the different materials of artificial femoral head and acetabular cup lining, it can be divided into metal to metal, metal to polyethylene, ceramic to polyethylene, ceramic to ceramic, and so on. Hemiarthroplasty was reported for the first time in “Artificial Femoral Head Summary of Femoral Neck Fracture” published in 1963 in China. The prosthesis used was the Judette femoral head, made of polymethyl methacrylate. The excellent and good rate of treatment was 4/7 [38]. Total hip arthroplasty was reported for the first time in the reference material of Orthopaedic Trauma in 1975, and the surgical procedures of artificial joint were introduced in detail. After 80 years of continuous development and improvement, THA has been mastered by more and more orthopedic surgeons. More and more elderly patients with acetabular fracture choose artificial hip replacement to improve the life quality after operation [39].

6 RCT articles were included in the end. A total of 445 samples were analyzed by meta-analysis. All the six RCT literatures included in this meta-analysis reported the baseline status of patients, only 3 RCT mentioned “random assignment” without any explanation, and the rest did not mention “random” information. The five studies included all gave detailed intervention measures. The number and reasons of blind method and lost follow-up or withdrawal were not described in detail in 6 RCT articles. Through the meta-analysis excellent and good rate between the experimental group and the control group through 6 RCT studies, the heterogeneity test results were chi^2^ = 6.11, df = 4, *P* = 0.19 > 0.05, and *I*^2^ = 35%, without obvious heterogeneity at *Z* = 2.68 and *P* = 0.007. These results suggested that the total hip arthroplasty application has the same excellent rate as other surgical treatment methods, indicating that total hip arthroplasty has a significant effect on the treatment of elderly acetabular fractures. Through the meta-analysis hip-joint function score, the heterogeneity test results were chi^2^ = 56.16, df = 4, *P* < 0.00001, and *I*^2^ = 93%, with obvious heterogeneity. The great difference was discovered in the hip function score between total hip arthroplasty and other surgical methods, showing that total hip arthroplasty can greatly improve hip-joint function. Then, the incidence of hip complications between the experimental cases and the control cases was calculated by meta-analysis. The heterogeneity test results were chi^2^ = 3.17, df = 4, *P* = 0.53 > 0.05, and *I*^2^ = 0%, without remarkable heterogeneity at *Z* = 3.05 and *P* = 0.002. This demonstrated that a significant difference was observed in the complication incidence, indicating that total hip arthroplasty displayed a lower incidence of hip-joint functional complications. The same idea can be found in the study put forward by other scholars [40–42]. They have applied new methods in the study, and the conclusions drawn can also give some support to this study. There are some limitations in this study. First of all, the sample size of the references included in this study is small, and they all belong to single-center research; there is a certain deviation. In the future research, we will carry out a large sample of prospective studies and hopefully draw more valuable conclusions.

The article "Effects of Different Surgical Procedures on the Therapeutic Effects, Prognosis, and Major Complications of Acetabular Fractures in the Elderly of China: A Systematic Review and Meta-Analysis" was published in 2022. Journal: Comput Math Methods Med.

## 5. Conclusion

Total hip arthroplasty has a good prognosis and a low complication rate in the treatment of acetabular fractures in the elderly of China. However, more studies and longer follow-ups are needed to further validate the findings of this study.

## Figures and Tables

**Figure 1:** Risk of bias.

**Figure 2:** Risk of bias summary.

**Figure 3:** Forest plot of meta-analysis of excellent and good rate.

**Figure 4:** Forest plot of meta-analysis of hip-joint function score.

**Figure 5:** Forest plot of meta-analysis of incidence of complications.

**Table 1:** Basic characteristics of literature.

Include the literature	Year of publication	*N* (C/T)	Treatment method		Outcome index	Whether it is random or not	Whether it is blind or not
			T	C			
Zhao Fuwen	2021	23/23	Open reduction and fixation	Total hip arthroplasty	①②③	Yes	No
Zhang Yong	2012	30/31	Surface replacement of hip joint	Total hip arthroplasty	①②③	Yes	No
Wang Yong	2014	35/30	Open reduction and fixation	Total hip arthroplasty	①②③	Yes	No
Li Xiangxiang	2018	50/50	Hemiarthroplasty	Total hip arthroplasty	②③	No	No
Liu Zhengmin	2020	43/50	Open reduction and fixation	Total hip arthroplasty	①②③	No	No
Xie Min	2014	40/40	Conservative treatment	Total hip arthroplasty	①	No	No

Note: ①: excellent and good rate; ②: hip-joint function score; ③: incidence of complications.

## Data Availability

No data were used to support this study.
